# Security Evaluation of Financial and Insurance and Ruin Probability Analysis Integrating Deep Learning Models

**DOI:** 10.1155/2022/1857100

**Published:** 2022-06-08

**Authors:** Yang Yang

**Affiliations:** School of Finance and Information, Ningbo University of Finance & Economics, Zhejiang 315175, China

## Abstract

To ensure safe development of the financial and insurance industry and promote the continuous growth of the social economy, the theory and its role of deep learning are firstly analyzed. Secondly, the security of financial and insurance and bankruptcy probability are discussed. Finally, an analytical model of the security bankruptcy probability of financial and insurance is designed through a deep learning model, and the model is evaluated comprehensively. The research results manifest that first, the designed security evaluation of the financial and insurance industry based on the deep learning and bankruptcy probability analysis model not only has strong learning ability but also can effectively reduce its own calculation error through short-time learning. Then, by comparing with other models, it is found that the designed model has a stronger ability to control various errors than other models, and the overall error rate of the model can be reduced to about 20%. At last, the data training indicates that the model designed by the deep learning method can accurately and effectively predict the basic situation of the financial and insurance industry, the minimum error can reach 0, and the highest is only about 3. The research provides a technical reference for the development of the financial and insurance industry and contributes to the prosperity of the social economy.

## 1. Introduction

With the expansion of science and technology, machine learning (ML) has become one of the main technologies for processing various tasks. Deep learning (DL) technology, as a technology of machine learning, provides important technical support for the current blossom of various industries [1]. As one of the current main economic development channels, the financial and insurance industry provides significant support for the growth of the social economy, and its security evaluation and ruin probability analysis are the main development guarantees [2]. It is a vital breakthrough to conduct a security evaluation of financial and insurance and ruin probability analysis through DL models. Although this work has not been fully applied, many studies have provided technical support for it.

Laak et al. [3] pointed out that DL was a research field that had received much attention in recent years and played an important role in ML. If shallow learning is a wave of ML, then DL, as a new field of ML, will set off another wave of ML. DL can interpret external data by establishing and simulating the hierarchical structure of the human brain to extract features from low-level to high-level external input data [3]. Dong et al. [4] proposed that the goal of DL was to improve learners' higher-order abilities such as solving problems, higher-order thinking, autonomous learning, and knowledge innovation. The DL evaluation should be guided by the goals of DL, using surveys, tests, statistical analysis, and other methods to make value judgments on the process and results of DL and to reflect and revise the goals of DL [4]. Buele et al. [5] believed that, in financial and insurance, risk estimation and prevention was the critical issue. The ruin probability was a good representation of the risk of the insurance business [5]. Bajwa and Rashid [6] deemed that keeping the bottom line of no systemic financial risk was the fundamental principle of doing a good job in financial work in the new era. To ensure the safe and stable operation of the financial system, it is necessary to properly manage every level of risk prevention and control and accurately and effectively deal with the risks hidden in all aspects of financial services. The financial escort business is an important part of financial services, and the improvement of its security service capability is a significant force for maintaining financial security and social stability and helps to enhance the ability of the financial system to prevent risks [6]. In a word, although the above research provides the latest research content of the DL technology and studies the security evaluation and bankruptcy risk of enterprises through different methods, there is a lack of research on integrating advanced DL technology with the security evaluation and bankruptcy probability of enterprises. Therefore, this research is groundbreaking in this regard.

To sum up, firstly, the basic connotation of DL is discussed, and the working principle of the DL model is expounded. Secondly, the security evaluation and bankruptcy probability of financial insurance are summarized. Finally, based on DL technology, the prediction and evaluation model of the security evaluation of financial insurance and bankruptcy probability analysis is designed, and the model is trained. The innovation of the research is that, by the DL model, not only the security evaluation model of enterprises is designed but also the bankruptcy probability of the enterprise can be predicted through the model. It provides a technical reference for the pullulation of the financial and insurance industry.

## 2. DL and Security Evaluation of Enterprises

### 2.1. Related Theories Based on DL

DL is a further in-depth study of the shallow neural network, and artificial neural network (ANN) is the basis of both. ANN is an extensive and interconnected network composed of adaptive neuron models [7]. In the model composed of neurons, neurons can receive signals from countless other neurons, and the transmission channels of these signals are connected to networks with weights. The neuron compares the received signal with its own neuron information, that is, the neuron's threshold. Then, the function processing system is activated through the threshold, thereby promoting the stimulation of neurons to generate output signals and connecting many of the same neurons to form the final neural network (NN) [8]. The basic element shape of an NN is shown in Figure 1.

In Figure 1, *x*, *y*, and *z* represent input features, hidden features, and output features, respectively, and have the same meaning as the elements in the subsequent figures. The activation of one neuron can generate a data analysis result, and many neurons are connected to form a complete NN model and output the analysis result of the complete data. The NN technology was first produced in the 1950s and 1960s, and the simplest NN technology is the perceptron, which is essentially a feedforward NN structure, and this NN structure is also relatively common [9]. The perceptron consists of an input layer, an output layer, and a hidden layer. The hidden layer is located between the input layer and the output layer and is the most vital structure in the NN model [10]. And, the neurons of the hidden layer and the output layer have activation functions, also known as functional neurons. The function of the activation function is to add nonlinear elements to the NN structure. These nonlinear elements will weight and sum the input values from other neurons during the working process of the system and map the processing results to the output [11]. The learning process of the NN is to process the input data, train its own computing model, and continuously update the threshold of functional neurons, to update the connection weights between neurons to achieve the purpose of learning and strengthen its own model function [12]. The calculation process of the specific form of the NN is shown in Figure 2.

In Figure 2, the three structural layers of the NN model have their own functions, and neurons between different layers are connected to each other, but neurons between the same layers are not connected to each other. Until the 1980s, the emergence of multilayer perceptron provided important technical support for the strengthening of NN models. A multilayer perceptron is a perceptron with multiple hidden layers, and it is also an ANN with a forward structure. The multilayer network of the multilayer perceptron is all connected to each other, and all the neurons of each layer of the NN are connected to the neurons of the previous layer, and each node has nonlinear activation functional neuron [13]. The gap between the multilayer perceptron and the single-layer perceptron is that the multilayer perceptron has multiple hidden layers. The multiple hidden layers greatly improve the computing power of the NN model, so that the multilayer perceptron can complete a variety of complex nonlinear computing tasks. In addition to shallow learning, DLNN also has DL technology. DL technology is that the NN model can process complex data through a deep nonlinear network structure. The multilayer perceptron is a DL structure. The essence of DL is to build an ML model with multiple hidden layers and train the model with massive training data to obtain more data features, thereby improving the computing speed and accuracy of the model. Compared with shallow learning models, DL models usually have 5, 7, or more hidden layers, and the design of DL models highlights the significance of feature learning. That is, the learning features are converted into a new feature space through layer-by-layer transmission, to construct their own feature learning mechanism, which makes the prediction and classification process of the model much simpler [14].

The learning mechanism of DL is mainly divided into two parts. The first step is unsupervised learning from top to bottom, that is, starting from the bottom, using unidentifiable data to train parameters at each level. The biggest difference from supervised algorithms that train shallow neural networks is that this learning process of DL models is unsupervised learning. The structure of the deep neural network (DNN) model is shown in Figure 3.

In Figure 3, it indicates the structure of the three-layer network of the DNN model. The first input is a six-dimensional vector, two hidden layers, and a two-dimensional (2D) output vector. The output is a probability value, which represents the probability that the input sample belongs to two classes. Before unsupervised training, the system initializes the network parameters randomly and then optimizes the parameters layer by layer through training. The parameters of the NN structure are gradually approached to the data features to optimize the output eigenvalues. After the parameters of the first layer are optimized, the feature learning can continue upward, and only the first and second hidden layers of the original NN are retained. Then, an output layer is added after the second hidden layer, and the eigenvalues learned by the first layer are used as the input values of the second layer for training. The training parameters are obtained in the same way, to minimize the error of the training parameters and obtain the second expression of the input data. Although the feature learning process has been completed so far, in practical applications, the level of the DNN model is much more than this. Therefore, the learning of features is more accurate, and the output value is more accurate [15].

The second step of DNN model training is top-down supervised learning, that is, adding a classifier to the top layer of the trained model and then training it through the algorithm of the shallow neural network. That is, the features of the first layer training are used as the input features of the last layer for training, and then more accurate feature values are obtained after training. When the above two steps of training are completed, the second classification can be performed for probability output, and the calculation process of the DNN model is completed [16].

### 2.2. Security of Financial and Insurance and Analysis Method of Ruin Probability

Insurance is significant support for the financial industry, and the insurance industry is also an important part of the financial industry. Therefore, the definition of security of financial and insurance can be defined with reference to industrial security. Therefore, the security of the insurance industry can be understood as a process of taking appropriate control over financial and insurance under the premise of matching social and economic progress and effective supply in the context of global economic integration. The concept of security in the insurance industry can be understood from two aspects. On the one hand, there are two conditions that the insurance industry needs to meet. The first condition is that the security of the insurance industry is a dynamic process; the second condition is that the social and economic development of the insurance industry matches the effective supply. Because financial and insurance products are not necessary for daily life, they have great demand elasticity, and the insurance industry, as an important part of the financial industry, has the temptation of demand in services, so its demand in the market is not effective demand [17]. However, the development of the insurance industry still plays a vital role in the development of the social economy, so it is still necessary to conduct comprehensive research on the safety of the financial and insurance industry, to comprehensively ensure the sustainable development of the financial and insurance industry and provide important support for the evolution of the society. On the other hand, the security of the insurance industry is essentially reflected in the balance of supply and demand, that is, the balance between the user's demand and the actual supply. If this balance cannot be maintained, no matter how society controls it, the security of the insurance industry will also be threatened. The security of a country's insurance industry needs to match the international economic environment and the competitive environment to ensure its stable progress [18].

Security impacts in the insurance industry include environmental impacts, competitive impacts, and control impacts. The environment of the insurance industry mainly refers to the proportion of social security in social financial expenditure, the proportion of insurance companies' tax burden in their revenue, the level of financial subsidies for policy insurance types, per capita GDP, the proportion of bank premium income in total premiums, and the proportion of insurance funds invested in funds and the proportion of savings deposits in GDP and many other factors. These factors have an important impact on the safety and development of the financial and insurance industry. The safety competition index of the insurance industry includes the market structure, market behavior, and market performance of the insurance industry and other influencing factors. Overall, it is divided into market concentration, insurance density, insurance depth, reserve accumulation ratio, Gini coefficient, owner's equity ratio, asset profit rate, net asset profit rate, premium income profit rate, and surrender rate. The control index of the insurance industry includes several aspects such as foreign capital's control of the insurance industry market, foreign capital's control of the insurance industry equity, and foreign capital's control of the insurance industry area. Therefore, to evaluate the security of the insurance industry, it is necessary to comprehensively evaluate the environment, competition, and control of the insurance industry [19].

Bankruptcy theory is a general theory for operators and decision-makers to quantitatively analyze and predict risks. Under a series of realistic assumptions, it uses tools such as probability statistics and stochastic processes to build models of random risks in the insurance business and study the nature of the models. Then, quantitatively analyze the bankruptcy risk and provide theoretical and technical support for the insurer to carry out effective risk management and control in reality. The main research object of bankruptcy theory is the risk model. Because it comes from the feasibility study of insurance companies and has a wide range of practical backgrounds in the fields of insurance, finance, securities investment, and risk management, bankruptcy theory research has always been an important direction in the field of actuarial research [20].

### 2.3. Financial Security and Analysis Model of Ruin Probability under DL

Firstly, a critical indicator in the establishment of the model is the time series, that is, the security evaluation and ruin probability analysis of the financial and insurance industry needs to be established on the time series, and the model is established with time as the main basis. When analyzing financial markets, financial transaction data is usually abstractly represented as financial time series, which includes opening price, closing price, highest and lowest transaction price, and transaction volume. Meanwhile, financial time series is also an application field of time series, so it also needs to be analyzed through time series. The main research content of time series is to find a reasonable technical method to achieve the purpose of ignoring the small fluctuations of the time series and obtain the concept of data shape, and simultaneously, it can identify its corresponding time series patterns on different time scales [21]. Each piece of data in a time series is composed of time variables and data variables, so a time series *T* of length *n* is shown as follows:

(1) $$\begin{array}{c} T=\left\{\langle t_{1},x_{1}\rangle ,\langle t_{2},x_{2}\rangle ,\ldots ,\langle t_{n},x_{n}\rangle \right\}, \end{array}$$

where *t* represents the time variable and *x* means the data variable. The financial time series usually use year, month, day, week, etc., as the main unit, and the time interval is uniform and continuous, so the financial time series is expressed as

(2) $$\begin{array}{c} X=\left\{x_{1},x_{2},\ldots ,x_{n}\right\}. \end{array}$$

The meaning of the parameters is the same as the above equation. In the constructed DL model, data processing is mainly carried out in the hidden layer, and the output results of each neuron in the first hidden layer are

(3) $$\begin{array}{c} F_{1p}=f\left(\sum_{i=1}^{d}\omega_{ip}x_{i}+b_{p}\right). \end{array}$$

*p* and *i* denote the sequence in the first hidden layer, *ω*_*ip*_ expresses the connection weight between neuron *i* and *p*, *b* means the threshold of the neuron, and *f* refers to the nonlinear activation function. The calculation result of the second hidden layer is

(4) $$\begin{array}{c} F_{2q}=f\left(\sum_{i=1}^{p}v_{iq}F_{1i}+c_{q}\right). \end{array}$$

*q* and *i* represent the sequence of neurons in the second hidden layer, *v*_*iq*_ indicates the connection weight between neurons *i* and *q*, and *c* shows the threshold of the neuron. And so on, through the calculation of the hidden layer, the output of the model is mapped to the output layer for output, and the training of the model is mainly carried out by the autoencoder. Autoencoder (AE) is an algorithm that can realize unsupervised training. AE includes encoder and decoder. The calculation of the encoder is

(5) $$\begin{array}{c} y=f\left(Wx+b\right). \end{array}$$

*W* and *b* are the parameters of the encoder, *f* is the nonlinear activation function, *y* is the feature, and *x* is the input value, and the decoding calculation is performed through the reconstruction of *y* and *x*. The calculation is

(6) $$\begin{array}{c} x^{\prime }=f\left(W^{\prime }y+b\prime \right). \end{array}$$

*W*′ and *b*′ are the parameters of the decoder, and the rest are the same as the above equations. The security evaluation of the financial and insurance and analysis of ruin probability established by the DL model is shown in Figure 4.

In Figure 4, the multilevel analysis of the DL model can not only improve the prediction accuracy of the financial and insurance industry but also continuously update the parameters of the model through error analysis. Then, the calculation effect of the model is gradually improved, which provides important support for the development of the financial and insurance industry.

### 2.4. Description of the Data

The model is verified and analyzed through the data set. The dataset contains the lending club (LC) dataset, which is the 105M dataset of LC (an online loan platform in the US) credit loan data from 2007 to 2017. LC is a peer to peer (P2P) lending. Its profit model is as follows: provide loans to borrowers (borrowers can get loans more quickly than in banks), and provide projects for investors (investors can get higher rates of return than banks here) [22]. Instead of investing itself, it charges a fee for every successful transaction by helping investors and borrowers “blind date.” The dataset contains 8.87 million credit records with 75 fields of information. Thera Bank (TB) dataset, which covers data of 5,000 customers, has 14 fields, namely, customer ID, age, work experience, income, zip code, family size, monthly credit card spending amount, education level, mortgage, personal loan business, bank securities account, bank deposit account, bank online facility, and bank credit card. Bank Marketing (BM) dataset, which is a 922 KB dataset, contains 11162 pieces of data and 17 fields of information, that is, 11162 rows *∗* 17 columns. The filter key field information is 12. By comparing the financial insurance security (FIS) model with the multilayer perceptron (MLP) model, the back propagation (BP) model, and the stacked autoencoder (SAE) model, the comparison indicators are mean square error (MSE), root mean square error (RMSE), mean absolute error (MAE), and error rate (ER) values. And, the calculation of these indicators is as follows [23]:

(7) $$\begin{array}{c} \text{MSE}=\frac{1}{n}\sum_{i=1}^{n}{\left(T_{i}-P_{i}\right)}^{2}, \end{array}$$

(8) $$\begin{array}{c} \text{RMSE}=\sqrt{\frac{1}{n}\sum_{i=1}^{n}{\left(T_{i}-P_{i}\right)}^{2}}, \end{array}$$

(9) $$\begin{array}{c} \text{MAE}=\frac{1}{n}\sum_{i=1}^{n}\left|T_{i}-P_{i}\right|, \end{array}$$

(10) $$\begin{array}{c} \text{ER}=\frac{\sum \left\{1|{\text{Model}}_{P}\neq {\text{Model}}_{T}\right\}}{\sum \left\{1|{\text{Model}}_{P}=\;{\text{Model}}_{P}\right\}}\times 100\%. \end{array}$$

*T* means the true value of the prediction, *P* demonstrates the predicted value of the model, *n* represents the number of samples, and *i* expresses the sequence of calculation samples.

## 3. Security Evaluation of Financial and Insurance and Calculation of Ruin Probability

### 3.1. Evaluation of DL Models

By building a DL model to evaluate the insurance security of the financial industry and analyze the ruin probability of the financial and insurance industry, through the establishment of the model, the security evaluation and the analysis of the ruin probability are achieved. The validation results on the DL model are shown in Figure 5.

In Figure 5, after the model's learning rate verification and error analysis, it is found that the designed model has advantages in all aspects. The first is that the learning rate of the model keeps rising as the number of iterations of the model increases. When the number of iterations reaches 10,000, the learning rate of the model is also about 0.9, which shows that the learning ability of the model is very strong. Meanwhile, in the error verification of the model, as the number of iterations increases, the error of the model gradually decreases. When the number of iterations of the model reaches 10,000, the error of the model is infinitely close to zero.

### 3.2. Performance Evaluation of the Model

The security evaluation and ruin probability prediction analysis of financial and insurance are the main basis for the financial industry to maintain stable or sustainable development. First, the prediction and evaluation model FIS is designed, and the specific performance of the designed model is tested by comparing with the models MLP, BP, and SAE. The comparison results between the designed model and other models are shown in Figure 6.

In Figure 6, the performance of different models is compared under different iterations. It indicates from the comparison results that the designed FIS model has the lowest error results under different iterations. Therefore, it can be seen that the designed model has better performance than the models MLP, BP, and SAE. And, the error rate of each model is also analyzed. The comparison results of the error rates of various models are shown in Figure 7.

In Figure 7, the error rate of each model is compared, and it is found that the error rate of the designed model is generally lower than that of other models. And, with the increase of the number of iterations, the error rate of the designed model decreases relatively more. When the number of iterations reaches 10,000, the error rate drops to about 21%. It denotes that the designed model performs better than the other models.

### 3.3. Analysis of the Safety of Financial and Insurance and Ruin Probability

Analysis of the safety of financial and insurance and ruin probability is the key to the survival of financial enterprises. Therefore, designing an effective model to predict the insurance safety and ruin probability of the financial industry is an important measure, which plays a decisive role in the development of the financial industry. So, a model is designed, different data sets are used to predict the financial industry index, and the prediction index used is the closing price of financial enterprises. The predicted results of the designed model are shown in Figure 8.

In Figure 8, the LC, TB, and BM data sets are used to predict the 100-day closing price of financial enterprises, and the specific performance of the designed model is analyzed by comparing it with the actual value. Through the analysis, it refers that the predicted results of the designed model in the three data sets are not much different, and the gap between the three error results is not large. Among them, the prediction error of the LC dataset is the lowest at about 0.2, and the highest is about 3; the prediction error of the TB dataset is at least 0 and the highest is about 2.5; the prediction error of the BM dataset is about 0 at the lowest and about 2.1 at the highest. It indicates that the designed prediction model can effectively predict the safety status and ruin probability of the financial and insurance industry and provide significant technical support for the development of the financial and insurance industry.

## 4. Conclusion

With the development of the times, more and more new start-ups emerge as the times require, but the increase in the number of new start-ups leads to a continuous decline in the survival probability of enterprises. Therefore, the security evaluation of enterprises and bankruptcy probability analysis are necessary means for current enterprise development. It mainly studies the security evaluation and bankruptcy probability analysis of the financial and insurance industry through DL models. It mainly designs and uses DL models and compares the designed model with other models to reflect the advantages of the designed model, and through data set training, the performance of the model can be evaluated. After research, firstly, it means that the designed model not only has strong learning ability but also can reduce the calculation error of the model through learning. Secondly, the performance of the designed model is superior to other models in many aspects, and through step-by-step data training, the error rate of the designed model can be quickly reduced to about 20%. Finally, the data set is used for model prediction training, and it is found that the designed model can better predict the transaction status of the financial and insurance industry, and the error is at least 0 and the highest is about 3. It illustrates that the designed model can effectively provide good forecast data and provide technical support for the progress of the financial and insurance industry. Although a complete model has been designed and comprehensively verified, in terms of research content, there is still a lack of specific factor analysis on the safety of the financial and insurance industry. Therefore, research in this area will be strengthened in the future to contribute to the development of the financial and insurance industry.

## Figures and Tables

**Figure 1:** Basic structure of NN. (a) The overall structure of the NN. (b) The calculation process of the structure of NN.

**Figure 2:** The specific structure of the NN model. (a) The overall structure of the NN model. (b) The calculation process of the first layer of the hidden layer and (c) the calculation process of the second layer of the hidden layer.

**Figure 3:** The structure of the DNN model.

**Figure 4:** The security evaluation of the financial and insurance and analysis of ruin probability established by the DL.

**Figure 5:** Verification results of the FIS model. (a) The verification result of the learning rate of the model in the hidden layer. (b) The analysis error verification of the model in the hidden layer.

**Figure 6:** Performance evaluation of the model. The model with (a) 1000 iterations, (b) 2000 iterations, (c) 3000 iterations, and (d) 4000 iterations.

**Figure 7:** Comparison results of model error rates. (a) The error rate analysis of various models. (b) The error rate analysis of each level of the FIS model.

**Figure 8:** The assessment results of insurance safety and ruin probability in the financial industry (a, c, e) are the comparison between the prediction results and the actual values using the LC, TB, and BM data sets, respectively; (b), (d), and (f) are the errors of the prediction results of the three data sets, respectively.

## Data Availability

All data are fully available without restriction.
